The article "Identification of the Novel Methylated Genes' Signature to Predict Prognosis in INRG High-Risk Neuroblastomas" was retracted in 2022. Reason: concerns about the peer review.

# Identification of the Novel Methylated Genes' Signature to Predict Prognosis in INRG High-Risk Neuroblastomas

**DOI:** 10.1155/2021/1615201

**Published:** 2021-09-13

**Authors:** Zhichao Liu, Changchun Li

**Affiliations:** Department of Surgical Oncology, Children's Hospital of Chongqing Medical University, National Clinical Research Center for Child Health and Disorders, Ministry of Education Key Laboratory of Child Development and Disorders;Chongqing Key Laboratory of Pediatrics, Children's Hospital of Chongqing Medical University, 136 Zhongshan 2nd Road, Yuzhong District, Chongqing 400014, China

## Abstract

**Background:**

Neuroblastomas are the most frequent extracranial pediatric solid tumors. The prognosis of children with high-risk neuroblastomas has remained poor in the past decade. A powerful signature is required to identify factors associated with prognosis and improved treatment selection. Here, we identified a strong methylation signature that favored the earlier diagnosis of neuroblastoma in patients.

**Methods:**

Gene methylation (GM) data of neuroblastoma patients from the Therapeutically Applicable Research to Generate Effective Treatments (TARGET) were analyzed using a multivariate Cox regression analysis (MCRA) and univariate Cox proportional hazards regression analysis (UCPHRA).

**Results:**

The methylated genes' signature consisting of eight genes (NBEA, DDX28, TMED8, LOC151174, EFNB2, GHRHR, MIMT1, and SLC29A3) was selected. The signature divided patients into low- and high-risk categories, with statistically significant survival rates (median survival time: 25.08 vs. >128.80 months, log-rank test, *P* < 0.001) in the training group, and the validation of the signature's risk stratification ability was carried out in the test group (log-rank test, *P* < 0.01, median survival time: 30.48 vs. >120.36 months). The methylated genes' signature was found to be an independent predictive factor for neuroblastoma by MCRA. Functional enrichment analysis suggested that these methylated genes were related to butanoate metabolism, beta-alanine metabolism, and glutamate metabolism, all playing different significant roles in the process of energy metabolism in neuroblastomas.

**Conclusions:**

The set of eight methylated genes could be used as a new predictive and prognostic signature for patients with INRG high-risk neuroblastomas, thus assisting in treatment, drug development, and predicting survival.

## 1. Introduction

Neuroblastomas are peripheral sympathetic nervous system embryonic tumors that arise from embryonic cells that make up the basic neural crest. Extracranial solid tumors are the most common neuroblastomas in children and responsible for up to 15% of cancer-related deaths [1–3]. The clinical course of neuroblastomas constitutes the progression of a complex heterogeneous disease. Localized neuroblastomas (stages L1 and L2), metastatic neuroblastomas (M), and metastatic neuroblastomas with specific characteristics in children younger than 18 months (MS) are the three types of tumors classified by the International Neuroblastoma Risk Group (INRG) [4, 5]. These risk markers (histology, age, MYCN, INRG stage, ploidy status, and 11q aberration) are used to divide patients into four pretreatment risk groups. There are three levels of difficulty: low, moderate, and high [6]. The low and intermediate groups show greater than 90% five-year survival rates, while the survival of the high-risk group remains poor at approximately 40%. Although advanced treatment consisting of surgery, chemotherapy, radiotherapy, and immunotherapy can be used in the course of treatment, all these have a poor survival rate for high-risk neuroblastomas [7]. This low prognosis needs the development of novel targeted medicines to improve the survival rate of high-risk neuroblastoma patients.

DNA methylation of CpG dinucleotides at gene promoter regions is a major regulatory mechanism involved in cellular processes that does not alter the DNA sequence [8]. DNA methylation reveals the pathogenesis and clinical behavior of neuroblastomas [9]. The most described DNA methylation alterations in neuroblastomas are CASP8 and RASSF1A [10, 11], and both are correlated with risk factors, such as age at diagnosis, MYCN amplification, and tumor stage [12–15]. Additionally, DNA hypomethylation of genes (CCND1, SPRR3, BTC, EGF, and FGF6) affects biological functions and pathogenesis in neuroblastomas [16]. In metastatic neuroblastomas, the hypermethylation status of TDGF1 and RB1 is associated with shorter survival, and genome-wide methylation profiling discovered novel methylated genes (PCDHGA4, TERT, DLX6-AS1, and DLX5) [17, 18]. However, epigenetic biomarkers for neuroblastomas are still very low. In particular, there are fewer methylation biomarkers associated with high-risk neuroblastoma patients.

In the current report, we identified significant and independent methylation prognostic biomarkers in INRG high-risk neuroblastomas from the TARGET database using phrase machine learning methods. The biomarkers could be used to design new therapy regimens for patients with high-risk neuroblastomas, potentially improving existing survival rates.

## 2. Materials and Methods

### 2.1. Retrieval of DNA Methylation Data for Analysis

Illumina HumanMethylation450 (Illumina Inc., California, USA) platform was used to evaluate DNA methylation data. There were 482,421 CpG sites on the methylation arrays throughout the genome [19], and each gene's overall beta value was represented by probe-level data. The TARGET data portal provided us with level 3 methylation data. We received 130 samples from the TARGET database, which contained DNA methylation data as well as clinical data such as gender, age, MYCN status, and INSS stage. All neuroblastoma samples are typically divided into two groups: training (86 cases) and testing (44 cases).

### 2.2. Construction of a Methylated Gene Signature in the Training Dataset

Hu et al. reported the best methods to construct signatures, and we used this approach for our study [20]. To begin, we used a UCPHR analysis to see if there was a link between survival rates and gene methylation in the training dataset [21]. The random survival forest-variable hunting (RSFVH) algorithm was then used to filter methylation genes, with ten being ruled out [22, 23]. For screening of predictive prognostic methylation genes, MCR analysis was utilized for constructing a model that could estimate the prognosis risk in accordance with the following expression:

(1) $$\begin{array}{c} \text{risk score}\left(\text{RS}\right)=\sum_{i=1}^{N}{\text{Meth}}_{i}*{\text{Coef}}_{i}. \end{array}$$

Here, the methylated genes of signature are represented by *N*, the value of methylation of the signature genes is represented by Meth_*i*_, while single CRO is denoted by Coef_*i*_. The multinode weighted sum of risk scores is known as the risk score (RS).

### 2.3. Statistical Analysis

A risk model was built using the aforementioned methylation gene signature. As a cutoff number, the median risk score was used for dividing the training and test patients into high-risk and low-risk groups [24]. Next, the ROC analysis and Kaplan–Meier survival (KMS) analysis were used to confirm the methylation gene signature's effective prognostic abilities in the test dataset. MCR analysis was used to determine the signature's independence in survival prediction, and a significant *P* value was less than 0.05. All analyses used the R program (version 3.5.1). Downloading of the randomForestSRC and pROC survival was carried out from Bioconductor (https://bioconductor.org).

### 2.4. Functional Analysis of the Signature of Methylated Genes

The DAVID bioinformatics tool was employed for predicting the activities of the signature of methylation genes using gene ontology (GO) analysis, which covered molecular functions, cellular components, and biological processes, as well as KEGG pathway enrichment studies (https://david.ncifcrf.gov/,version 6.8). The value of *P* < 0.05 is considered significant for GO and KEGG pathways.

## 3. Results

### 3.1. Clinical Characteristics' Analysis of TARGET Data

All of the expression data used in this investigation came from patients with neuroblastomas, both clinically and pathologically. We conducted a statistical analysis of the clinical data (gender, age, MYCN status, and INSS stage) in the test group and training group. The results revealed high-risk patients had only occupied no more than 5% <18 months and included 97.7% INSS stage 4 in the test group and training group. The details of clinical/pathological features can be found in Table 1. After that, the 130 patients were randomly separated into two groups (test group, *n* = 44; training group, *n* = 86) to examine if the methylation genes revealed in neuroblastoma patients had any prognostic significance.  Figure 1 shows the selection process for the methylated genes' signature.

### 3.2. Construction of the Survival Methylated Genes' Signature

The training group (*n* = 86) with all clinical data was used to investigate the relationship between overall survival and the presence of methylated genes. We first performed a univariate CPHR analysis of the methylation genes' profiling data with survival status and survival time as dependent factors. We discovered 339 methylation genes that were significantly linked to the patient's overall survival (*P* value <0.05, Figure 2). The 339 genes were then analyzed using the random forest technique to evaluate the signature of methylation genes. Based on their permutation importance score (PFI) using the RSFVH method, the analysis found ten genes that were substantially linked with patient overall survival (Figure S1).

We utilized a CMR analysis (Table S1) to develop an eight-methylation gene set model (NBEA, DDX28, TMED8, LOC151174, EFNB2, GHRHR, MIMT1, and SLC29A3) for assessing the risk to survival for screening the most powerful, predictive, prognostic methylated genes. The risk scores (Table S2) of the combination which composed NBEA, DDX28, TMED8, LOC151174, EFNB2, GHRHR, MIMT1, and SLC29A3 were determined as follows:

(2) $$\begin{array}{c} \text{RS}=\left(-3.65\times {\text{meth}}_{\text{NBEA}}\right)+\left(-22.66\times {\text{meth}}_{\text{DDX}28}\right)+\left(20.60\times {\text{meth}}_{\text{TMED}8}\right)\\ +\left(-6.13\times {\text{meth}}_{\text{LOC}151174}\right)+\left(8.48\times {\text{meth}}_{\text{EFNB}2}\right)\\ +\left(0.01\times {\text{meth}}_{\text{GHRHR}}\right)+\left(-4.11\times {\text{meth}}_{\text{MIMT}1}\right)+\left(20.43\times {\text{meth}}_{\text{SLC}29\text{A}3}\right). \end{array}$$

Here, risk score is denoted by RS, while the values of methylation are denoted by meth.

### 3.3. Determining the Survival Power of the Methylated Genes' Signature in the Training and Test Dataset

For each patient, the analysis gave a risk score for the identified methylation genes' signature. Using the median risk score, we divided the training group into two groups: low risk (*n* = 43) and high risk (*n* = 43). Using the Kaplan–Meier survival (KMS) analysis, it was observed that the high-risk group had considerably lower survival rates than the low-risk group (median survival time: 25.08 months vs. >128.80 months, log-rank test, *P* < 0.001; Figure 3(a)). The high-risk group had a 5-year survival rate of fewer than 20%, while the low-risk group had a rate of more than 60%. The risk scores based on the methylation genes' signature of the test group patients were calculated using the same prognostic risk score methodology, confirming the predictive value of the signature. Similarly, the two risk groups in the test dataset were displayed using Kaplan–Meier curves (Figure 3(b)). The high-risk group in the study had a significantly lower median survival time than the low-risk group (median survival time: 30.48 months vs. >120.36 months, log-rank test, *P* < 0.01). The high-risk group had a survival rate of less than 30%, whereas the low-risk group had a survival rate of more than 50%.

### 3.4. The Survival Prediction Power of the Methylated Gene Signature in the Test and Training Groups

ROC analysis was used to assess the methylation gene signature's predictive capacity, with the higher area under the ROC curve indicating a better model for neuroblastoma patients' expected survival. The eight methylated gene signatures had a strong prediction ability in the training group (AUC_Signature_ = 0.87, Figure 3(c)), indicating that the methylated gene signature in the present study was a highly accurate novel survival biomarker. A similar highly accurate result was also observed in the test group (AUC_Signature_ = 0.71, Figure 3(d)). The DNA methylation level of each gene in the training dataset has been compared with a *t*-test (Table S3). The distribution of the DNA methylation level of each of the eight genes in the total group (*N* = 130) was analyzed (Figure 4). Most genes except GHRHR showed significant differences in methylation levels between the low- and high-risk groups.

### 3.5. The Selected Eight Methylated Genes' Signature Is an Independent Prognostic Factor

We used a MCR analysis, which included the risk scores based on the signature as well as various clinical characteristics (such as gender, age, MYCN status, and INSS stage). This analysis was utilized to show the prognostic efficacy of the methylated genes' signature risk score for overall survival prediction, which was an independent prognostic factor across all datasets (high-risk dataset vs. low-risk dataset, HR = 2.13, 95% CI: 1.70–2.66, *P* < 0.001, *n* = 194, Table 2).

### 3.6. Functional Analysis of the Methylated Genes' Signature

GO and KEGG analyses were employed for investigating these DNA methylation genes' potential involvement in biological processes associated with neuroblastoma development (Figure 5, Table S4). Results showed that eight methylated genes were involved in butanoate metabolism, beta-alanine metabolism, propanoate metabolism, glutamate metabolism, and tryptophan metabolism, which are all associated with energy metabolism. It was reported that neuroblastoma cells were strictly dependent on glucose metabolism, which has been discovered to be a very frequent feature among tumors that are otherwise biologically diverse. In addition, glycolysis intermediates are key precursors for cell growth in addition to generating ATP [25]. As a result, the modulation of these genes by methylation played various important roles in the process of energy metabolism in neuroblastomas.

## 4. Discussion

Neuroblastomas are the most prevalent extracranial pediatric solid tumors responsible for a disproportionate amount of pediatric cancer mortality. They arise in the developing sympathetic nervous system [26, 27]. Although there have been advances in therapies for patients, some of which include myeloablative chemotherapy and intensive induction chemotherapy, the overall outcome for high-risk neuroblastoma patients is still unacceptably poor [28]. Three recent studies focused on prognosis in neuroblastoma. An 18-gene signature predicted the clinical outcome in stage 4 neuroblastoma [29] and found ERCC6L, AHCY, STK33, and NCAN as a set of genes that could be used to predict prognosis in neuroblastoma patients [30]. MELK was a novel therapeutic target for high-risk neuroblastomas [31]. However, methylation gene signatures and their relationship to neuroblastoma survival have been studied infrequently, particularly in high-risk individuals. We employed a combination of phrase machine learning methods and statistical methodologies to establish a methylation genes' signature composed of ten genes in our investigation. They were found to be relevant to the survival of patients with neuroblastomas. Using gender, age, MYCN status, and INSS stage as covariables, the independence of the chosen signature in survival prediction of neuroblastoma patients was evaluated using an MCR analysis. The signature-based risk scores of patients were found to be independently associated with overall survival. As a result, we found that the methylated genes' signature predicted independently in patient overall survival. These findings showed that the predictive value of the methylation genes' profile for predicting survival of neuroblastoma patients had no response for other clinical factors.

After a variety of analyses, eight significant gene methylation events were identified. EFNB is a member of the Eph family receptor tyrosine kinases, and reports have shown that EFNB2 is regulated and can perform prognostic roles in neuroblastomas. For example, high-level expression of transcripts encoding EPHB6 receptors (in association with their ligands EFNB2 and EFNB3) was predictive of neuroblastoma [32], and EFNB2 was induced by WNT signaling. As a result, EFNB is likely to have a role in neuronal development and neuroblastoma cell fate decisions [33]. Previous studies also suggested that there are many potential associations between diseases and EFNB2. One such example was demonstrated when it was found that microRNA-137 inhibited EFNB2 expression affected by a genetic variant in schizophrenia patients [34]. Starting in midgestation, NBEA encoded a member of a broad, diversified set of A-kinase anchor proteins that was substantially expressed in the mouse brain [35, 36], and this expression affected postsynaptic neurotransmitter receptor trafficking to the cell surface [36, 37]. Studies have demonstrated that NBEA not only was a predicted signature [38–40] but also played an important regulatory role in neurodevelopment [41, 42]. NBEA has been shown to act as a gene signature to predict the prognosis of gastric cancer [43] and as a transcriptional regulator in the nucleus, where it interacts with NOTCH1. This association was found particularly important for pathogenesis as NOTCH signaling is required for brain development [44]. GHRHR is the growth hormone-releasing hormone receptor gene. Overexpression of GHRHR has been shown to have an oncogenic role associated with several types of cancers, including neuroblastoma [45]. SLC29A3 encodes a nucleoside transporter which plays a significant role in the cellular uptake of nucleosides and nucleobases. It was previously reported that many diseases were related to RAD51AP1 expression, including autoinflammatory diseases [46], H syndrome [47], insulin-dependent diabetes [48], pigmentary hypertrichosis, autoimmune insulin-dependent diabetes mellitus [49], and sclerosing bone dysplasias [50]. Meanwhile, MIMT1 is an MER1 repeat-containing imprinted transcript, which can undergo hypermethylation in the placenta of intrauterine growth-restricted fetuses in cattle [51], and truncation of exons 3 and 4 of the MIMT1 gene caused intrauterine growth restriction [52]. Furthermore, the transmembrane p24 trafficking protein family member, DDX28, was used to investigate pediatric-onset genetic disorders by digital PCR [53]. However, the biological roles of the two genes (TMED and LOC151174) in cancer are yet unknown, and this has to be researched further in future research. These previous studies demonstrate that the signature outlined in the current work can predict prognostic outcomes and inform clinical treatment.

In terms of neuroblastomas, there are a few drawbacks to this study. Most importantly, more studies into the specific mechanism of gene methylation in neuroblastomas are needed. Furthermore, the methylation genes' signature is yet to be tested in clinical trials. Even after these limitations, the continuous and significant corelation of our methylation genes' signature with overall survival in two separate groups suggested that it could be a useful and powerful predictive signature for neuroblastomas.

The use of phrase machine learning has allowed us to identify a methylated genes' signature which provided more clinically significant prediction accuracy.

## Figures and Tables

**Figure 1:** The research flowchart. The sequence of analyses for developing the RC model and validating the signature's ability to predict prognostic outcomes.

**Figure 2:** Identification of the methylated genes' signature in the training dataset. UCPHRA of the gene methylation profiling data in the training dataset used to predict the methylated genes' signature in the test and training datasets.

**Figure 3:** Patients with neuroblastoma have a methylated gene signature that predicts overall survival. (a) KMS curves were used for dividing the patients into high- and low-risk groups. Log-rank tests were used to calculate *P* values. (b) Results of receiver operating characteristic (ROC) analysis.

**Figure 4:** The distribution of the DNA methylation level of each of the eight genes between high- and low-risk groups in the total group (*N* = 130).

**Figure 5:** Functional enrichment of the eight methylated genes' signature. (a) Gene ontology (GO) plot displaying gene ratios for the eight methylated genes' signature. (b) KEGG analysis of the 8 methylated genes' signature.

**Table 1:** Summary of patient characteristics and demographics.

Characteristic	Number of cases (%) in the training set	Number of cases (%) in the testing set
*Gender*		
Male	47 (54.7%)	29 (82.6%)
Female	39 (45.3%)	15 (17.4%)
*Age*		
<18 months	2 (2.3%)	2 (2.3%)
≥18 months	86 (97.7%)	42 (97.7%)
*MYCN status*		
Amplified	31 (36.0%)	17 (38.6%)
Not amplified	54 (62.8%)	27 (61.4%)
NA	1 (1.2%)	
*INSS stage*		
1	0 (0.0%)	0 (0.0%)
2	0 (0.0%)	0 (0.0%)
3	2 (2.3%)	0 (0.0%)
4	84 (97.7%)	43 (97.7%)
4s	0 (0.0%)	1 (2.3%)
*INRG*		
Low risk	0 (0.0%)	0 (0.0%)
Intermediate risk	0 (0.0%)	0 (0.0%)
High risk	89 (100%)	44 (100%)
*Vital status*		
Living	35 (40.7%)	20 (55.5%)
Dead	51 (59.3%)	24 (54.5%)

**Table 2:** Univariable and multivariable Cox regression analyses of the association between the eight methylated genes' signature and the survival of neuroblastoma patients in the total group (*n* = 130).

Variables		HR	95% CI of HR		*P*
			Lower	Upper	
*Univariable analysis*					
Gender	Male vs. female	1.17	0.73	1.87	0.52
Age	>18 months vs. ≤18	0.97	0.90	1.06	0.51
MYCN status	Amplified vs. non	1.24	0.77	1.98	0.38
Methylated genes' signature	High risk vs. low risk	2.02	1.65	2.47	≤0.001
*Multivariable analysis*					
Gender	Male vs. female	0.89	0.55	1.44	0.64
Age	>18 months vs. ≤18	1.01	0.93	1.11	0.79
MYCN status	Amplified vs. non	0.77	0.46	1.30	0.33
Methylated genes' signature	High risk vs. low risk	2.13	1.70	2.66	≤0.001

## Data Availability

All the data used to support the findings of this study are included within the article and are available at The Cancer Genome Atlas (TCGA) database.

## Supplementary Materials

Supplementary Materials Figure S1: random survival forest-variable hunting analysis reveals the error rate for the data as a function of trees. Table S1: methylated genes of univariate Cox regression analysis (*P* < 0.05) in the training set (*n* = 86). Table S2: multivariate Cox regression analysis of the 8 methylated genes and survival of neuroblastomas patients in the training group. Table S3: the signature risk score composed of 8 combinations in the training and test dataset. Table S4: different DNA methylation genes between the high- and low-risk groups. Table S5: functional enrichment of the 8 methylated genes' signature.
